# Effect of Human-Oriented Fine Nursing on Psychological Emotion, Life Quality, and Nursing Satisfaction of Patients Undergoing Laparoscopic Radical Nephrectomy

**DOI:** 10.1155/2022/5016967

**Published:** 2022-08-08

**Authors:** Hong Yu, Wei Dong

**Affiliations:** ^1^Department of Urinary Surgery, Sheng Jing Hospital of China Medical University, Shenyang, Liaoning, China; ^2^Department of Pathology, Weifang Traditional Chinese Hospital, Weifang, Shandong, China

## Abstract

**Purpose:**

This study set out to explore the therapeutic effects of human-oriented fine nursing intervention on patients undergoing laparoscopic radical nephrectomy and its influence on patients' quality of life.

**Methods:**

A total of 120 patients who underwent laparoscopic radical nephrectomy in Sheng Jing Hospital of China Medical University from January 2019 to January 2020 were randomized into group A (*n* = 60) and group B (*n* = 60) by the random table method. Group B was treated with routine nursing while group A was additionally treated with human-oriented fine nursing. Meanwhile, the study compared the two groups in terms of vital signs, postoperative recovery time, visual analogue scale (VAS), sleep quality (SQ), adverse psychological response score, and quality of life (QOL).

**Results:**

According to our findings, patients of group A had significantly lower heart rate, blood pressure, and adverse psychological response scores compared to those of group B; the postoperative recovery time of group A was considerably shorter than that of group B; the VAS scores of group A at 3 and 6 days after surgery were markedly lower than those of group B; group A had a remarkably higher number of patients with excellent postoperative SQ than group B; and group A saw substantially higher QOL scores of patients compared to group B.

**Conclusion:**

Results of this study suggested that fine nursing intervention based on humanistic care for patients undergoing laparoscopic radical nephrectomy can improve the physical condition of patients, refine their mentalities, and improve their sleep quality, thus enhancing their quality of life and accelerating the recovery process. Therefore, this nursing mode is worthy of promotion and application in clinical practice.

## 1. Introduction

Renal cell carcinoma is one of the most common malignant tumors in the urinary system [1]. It is a malignant tumor originating from the renal parenchymal urinary tubule epithelial system, also known as renal adenocarcinoma, accounting for 80% ∼ 90% of renal malignant tumors [2]. Advanced renal cancer is mainly treated by surgical resection of tumor lesions combined with biological therapy, endocrine therapy, and immunotherapy, which is not effective and patients are prone to intolerance [3]. Based on the holistic view and syndrome differentiation, traditional Chinese medicine believes that renal cell cancer is caused by deficiency of kidney qi and aggregation of pathogenic toxins [4]. The application of TCM treatment can improve the healthy qi, stabilize the cancer focus, prevent recurrence and metastasis, and thus achieve the purpose of improving the quality of life of patients and prolonging their survival [5, 6].

Currently, laparoscopic radical nephrectomy is the preferred measure for the treatment of renal carcinoma by virtue of its minimally invasive approach and small incision, which theoretically can accelerate the postoperative recovery and improve the effects of functional rehabilitation [7]. Nonetheless, previous studies on patients undergoing laparoscopic radical nephrectomy show that adverse psychological responses and body aches or pains affect the overall therapeutic efficacy to a certain extent, which underlines the necessity of comprehensive and efficient fine nursing to improve surgical effects [8, 9]. In general, fine nursing refers to treatment striving for excellence throughout the whole process of nursing implementation, systematically optimizing and upgrading previous nursing measures so as to enhance the quality and efficiency of nursing and further provide more quality nursing to patients [10]. Moreover, to give full play to the human-oriented thought of nursing discipline, nursing staff should take the humanistic care concept as the operating principle and implement Nightingale's spirit in the implementation of fine nursing to improve patients' mentalities and quality of life [11, 12]. Based on this, the study aimed to investigate the impact of human-oriented fine nursing intervention on patients undergoing laparoscopic radical nephrectomy. It selected 120 eligible inpatients admitted from January 2019 to January 2020 as the subjects, and the research results are as follows.

## 2. Materials and Methods

### 2.1. General Information

This study was a prospective randomized-controlled study. It could not set enrollment blind to the intervention method. So, the data collector and data analyst were blind in this study, and the enrollments were informed of the intervention method. A total of 120 patients who underwent laparoscopic radical nephrectomy in Sheng Jing Hospital of China Medical University from January 2019 to January 2020 were randomized into group A (*n* = 60) and group B (*n* = 60) by the random table method. During the recruitment phase, neither the researchers nor the physicians had access to the randomization list. This study has been permitted by the ethics committee of China Medical University (no. 2019/29–494).

### 2.2. Inclusion Criteria

(1) All participants and their families were informed about the details of the research and signed the informed consent form before the enrollment; (2) patients were diagnosed with renal cancer and had undergone laparoscopic radical nephrectomy; and (3) age 18∼80 years old.

### 2.3. Exclusion Criteria

(1) Those with lymph node metastasis or venous cancer thrombus; (2) those had mental problems or were unable to conduct communication; and (3) those who suffered from other organic diseases.

### 2.4. Methods

Group B was treated with routine nursing, and the specific measures were as follows: (1) nursing staff conducted the perioperative nursing according to the doctor's advice. They observed the patient's signs data to timely determine if any deterioration has occurred; (2) nursing staff provided analgesic drugs to patients when necessary and preoperative psychological counseling to relieve their negative mood; (3) nursing staff ensured that patients were in an appropriate position and kept watching whether the drainage tube was working well.

In the meantime, Group A was treated with fine nursing based on humanistic care besides conventional nursing, and the specific measures were as follows: (1) preoperative psychological nursing: nursing staff knew the patients' information in detail and developed nursing plans according to patients' individual conditions; they also informed patients before the operation of knowledge on the disease, the surgery, and pain, so that patients understood the advantages of laparoscopic surgery and what they might face after the operation; when communicating with patients, nursing staff should listen to patients' demands, ask them about their worries, and propose corresponding treatment measures according to their specific issues, so as to help them express tension and relentlessness. (2) Basic preoperative care: a quality control group was set up to summarize and analyze the problems in the previous care and put forward improvement plans; the nursing staff should arrange the patient to have a routine examination on the day of operation and submit the examination results; they assisted with surgery preparation of patients, such as shaving, stop eating for 12 hours, and drinking for 6 hours before surgery to ensure clean intestines. (3) Postoperative psychological care: nursing staff informed the patient's family members about what the patient was facing and guided them to keep a close eye on the patient's expression to determine whether he or she was in pain, and thereby take the appropriate pain-relieving measures; nursing staff asked patients about their feelings after surgery, informed them of pain relief methods, and played music for them; they established narrative connection with patients, put themselves in the position of patients, increasing their own empathy and appreciating the will of patients. (4) Basic postoperative care: nursing staff should tell whether the patient had acidosis, and do a good job of catheter care and drainage tube care; they kept patients to maintain in a comfortable and correct position, carried out diet intervention; they encouraged patients to get out of bed and exercise as soon as possible, and conducted appropriate exercise intervention for them.

### 2.5. Observation Criteria

1. Comparison of patients' vital signs: heart rate, systolic blood pressure, and diastolic blood pressure before and after surgery were measured and recorded in the two groups.
2. Comparison of postoperative recovery time, including time of anal exhaust, extraction time of drainage tube, time of getting out of bed, and wound healing.
3. Comparison of patients' VAS scores [13]: VAS scores at 1 day (T1), 3 days (T2), and 6 days (T3) after surgery were recorded, ranging from 0 to 10 points. The rising of the score manifested that the pain became more and more intense.
4. Comparison of postoperative SQ: the SQ of patients was evaluated by the self-designed scale of our hospital. Patients were considered to have excellent sleep quality when they had an average sleep time of over 8 hours per day and no drowsiness or irritation in the daytime; those who had good sleep quality when they had a sleep time of between 5 hours and 8 hours per day and no obvious sleepiness or irritability in the daytime; and those had poor sleep quality when they slept less than 5 hours a day with obvious drowsiness or restlessness in the daytime. The number of patients with the above-mentioned different SQ was respectively counted and the proportion was calculated.
5. Comparison of adverse psychological response [14]: the study employed the Self-Rating Depression Scale (SDS) and Self-Rating Anxiety Scale (SAS) in the hospital. It showed that the score rose in accordance with the degree of seriousness of adverse psychological response.
6. Comparison of QOL after nursing [15]: based on the QOL-C30 quality of life scale, the study compared the two groups on aspects of patients' scores of emotional function, cognitive function, role function, physical function, and social function. A lower score corresponded to worse QOL.

### 2.6. Statistics

The statistical analysis was conducted with SPSS 20.0 software and Graphics drawing was carried out with GraphPad Prism 7 (GraphPad Software, San Diego, USA) in this study. Measurement data were represented as ($\bar{\text{x}}\pm \text{s}$) and analyzed by *t*-test. Enumeration data were represented as (*n*, %) and analyzed by the *χ*^2^ test. *P* < 0.05 indicated a statistically significant difference.

## 3. Results

### 3.1. Comparison of General Data

There was no significant difference in the general information of the two groups (*P* > 0.05), as shown in Table 1.

### 3.2. Comparison of Patients' Vital Signs

After nursing, significantly lower heart rate and blood pressure were observed in group A compared to group B (*P* < 0.001), as shown in Table 2.

### 3.3. Comparison of Postoperative Recovery Time

In contrast to group B, patients in group A needed considerably less time for postoperative recovery (*P* < 0.001), as shown in Table 3.

### 3.4. Comparison of VAS Scores

The VAS scores of group A at 3 days and 6 days after surgery were significantly lower than those of group B (*P* < 0.001), as shown in Figure 1.

### 3.5. Comparison of Postoperative SQ

The number of patients with excellent postoperative SQ in group A was remarkably higher than that in group B (*X*^2^ = 8.086, *P*=0.004), as shown in Table 4.

### 3.6. Comparison of Adverse Psychological Response Scores

Group A reported significantly lower scores of adverse psychological responses after nursing than group B (*P* < 0.001), as shown in Table 5.

### 3.7. Comparison of QOL after Nursing

QOL scores in group A were significantly higher than those in group B (*P* < 0.001), as shown in Table 6.

## 4. Discussion

It is well-known that laparoscopic radical nephrectomy can virtually reduce the operative time and facilitate recovery [16, 17]. However, patients still suffer from postoperative pain and adverse psychological responses, for which they may exhibit such symptoms as speeding of heart rate, a rise in blood pressure, or reduction of sleep quality, increasing the occurrence of complications to a certain extent [18]. Undoubtedly, quality perioperative nursing is a powerful measure to relieve patients' physical discomfort and negative mentalities [19]. In this study, patients in group A obviously outperformed patients in group B on the aspects of heart rate, blood pressure, and adverse psychological response scores after fine nursing (*P* < 0.001 and had significantly lower VAS scores at 3 and 6 days after surgery (*P* < 0.001), taking advantage of communication between patients who poured out their appeals and nursing staff who provided pain-relieving treatment according to patients' description of their pain and guided them to express bad feelings. Therefore, patients in group A exhibited better vital signs and suffered less pain.

Additionally, it was found that significantly more patients in group A obtained excellent and good SQ after surgery compared to group B (*P* < 0.05), and the QOL score of group A was significantly higher than that of group B (*P* < 0.001), for those patients in group A timely expressed negative emotions and had less physical pain disturbing their sleep. Furthermore, nursing staff increased the frequency of interaction with patients' family members and consequently gave patients bilateral care, improving their overall quality of life [20]. Owing to a better quality of life and physical condition, patients in group A needed less time for recovery after surgery compared to patients in group B (*P* < 0.001), suggesting that human-oriented fine nursing was beneficial to patients by speeding up the recovery process.

## 5. Conclusion

Human-oriented fine nursing for patients undergoing laparoscopic radical nephrectomy can improve the physical condition of patients, refine their mentalities, and improve their sleep quality, thus enhancing their quality of life and accelerating the recovery process. Therefore, this nursing mode is worthy of promotion and application in clinical practice.

## Figures and Tables

**Figure 1:** Comparison of VAS scores. Note: the horizontal axis represents 1 day (T1), 3 days (T2), and 6 days (T3) after surgery, and the vertical axis represents VAS scores (points). The VAS score at T1 was 3.2 ± 0.2 in group A and 3.2 ± 0.3 in group B. The VAS score at T2 was 2.1 ± 0.2 in group A and 2.6 ± 0.3 in group B. The VAS score at T3 was 1.0 ± 0.1) in group A and 1.5 ± 0.2 in group B. ^*∗∗∗*^*P* < 0.001.

**Table 1:** General data.

	Group A (*n* = 60)	Group B (*n* = 60)	*χ* ^2^/*t*	*P*
Gender (male/female)	40/20	41/19	0.038	0.845
Age (years)	46.2 ± 6.2	46.3 ± 6.1	0.089	0.929
Tumor size (cm)	4.2 ± 1.9	4.3 ± 2.0	0.281	0.779
Pathological type			0.044	0.835
Clear cell	45	44		
Papillary	15	16		

**Table 2:** Comparison of vital signs ($\bar{x}\pm s$).

	Heart rate (beats/min)		SBP (mmHg)		DBP (mmHg)	
	Before	After	Before	After	Before	After
Group A (*n* = 60)	75.1 ± 10.2	70.3 ± 9.5	117.2 ± 10.3	124.4 ± 10.5	72.1 ± 5.8	83.1 ± 4.6
Group B (*n* = 60)	75.2 ± 10.3	85.6 ± 9.7	117.5 ± 10.6	148.6 ± 12.3	72.2 ± 5.9	95.8 ± 4.5
*t*	0.053	8.729	0.157	11.591	0.094	15.287
*P*	0.958	<0.001	0.875	<0.001	0.926	<0.001

**Table 3:** Comparison of postoperative recovery time ($\bar{x}\pm s$).

	Anal exhaust (h)	Drainage tube extraction (h)	Getting out of bed (h)	Wound healing (d)
Group A (*n* = 60)	27.6 ± 3.2	53.2 ± 3.5	26.8 ± 4.1	7.8 ± 0.2
Group B (*n* = 60)	36.1 ± 3.2	61.2 ± 5.8	30.6 ± 3.8	8.5 ± 0.1
*t*	14.549	9.148	5.265	24.249
*P*	<0.001	<0.001	<0.001	<0.001

**Table 4:** Comparison of postoperative SQ (*n*, %).

	Excellent	Good	Poor	Excellent-to-good sleep rate
Group A (*n* = 60)	30	28	2	58 (50.00)
Group B (*n* = 60)	18	30	12	48 (36.00)
*χ* ^2^				8.086
*P*				0.004

**Table 5:** Comparison of adverse psychological response scores ($\bar{x}\pm s$, points).

	SDS		SAS	
	Before	After	Before	After
Group A (*n* = 60)	68.2 ± 10.2	35.4 ± 5.6	68.1 ± 11.2	37.1 ± 12.3
Group B (*n* = 60)	68.3 ± 11.0	45.2 ± 4.8	68.5 ± 11.0	48.2 ± 14.5
*t*	0.052	10.292	0.197	4.522
*P*	0.959	<0.001	0.844	<0.001

**Table 6:** Comparison of QOL after nursing.

	Emotional function	Cognitive function	Role function	Physical function	Social function
Group A (*n* = 60)	85.1 ± 4.2	75.2 ± 5.2	75.8 ± 3.2	78.6 ± 2.4	75.4 ± 6.5
Group B (*n* = 60)	74.2 ± 5.4	69.1 ± 3.4	65.2 ± 3.1	67.2 ± 3.6	67.2 ± 3.4
*t*	12.34	7.61	18.43	20.41	8.66
*P*	<0.001	<0.001	<0.001	<0.001	<0.001

## Data Availability

The datasets used during the present study are available from the corresponding author upon reasonable request.
